The article "Observation of Curative Effect of Lung Recruitment in Patients with Acute Respiratory Distress Syndrome after Cardiopulmonary Bypass Surgery" was retracted in 2023. Reasons: signs of a paper mill; suspected computer-generated content; unreliable results or conclusions; concerns about the data.

# Observation of Curative Effect of Lung Recruitment in Patients with Acute Respiratory Distress Syndrome after Cardiopulmonary Bypass Surgery

**DOI:** 10.1155/2022/2693500

**Published:** 2022-09-12

**Authors:** Lin Guo, Jinxiu Zeng, Ziyou Liu, Zijie Wei, Caiyun Wen, Yue Zhang, Xu Chen, Heping Xie

**Affiliations:** ^1^Cardiac ICU, First Affiliated Hospital of Gannan Medical College, Ganzhou, 341000 Jiangxi, China; ^2^Disinfection Supply Centers, First Affiliated Hospital of Gannan Medical College, Ganzhou, 341000 Jiangxi, China

## Abstract

Recruitment maneuver (RM) has become a routine supplementary maneuver for clinical rescue of severe ARDS with low tidal volume/pressure-limited mechanical ventilation. Recruitment of patients with ARDS mechanical ventilation can improve the lung compliance, promote the opening of collapsed alveoli, improve the ratio of ventilation to blood flow, reduce dead space, reduce shunt flow, and improve oxygenation function. In this paper, the patients were divided into lung recruitment group and conventional treatment group by the random number permutation table method. When the patient's percutaneous oxygen saturation is less than or equal to 88%, the partial pressure of oxygen in the arterial blood gas is less than or equal to 55 mmHg, or the ventilator tube is disconnected during sputum suction or other accidents, a CPAP × 60 − second lung recruitment maneuver is required. Then adjust the ventilator parameters in the same way. In the process of lung recruitment, the changes in invasive continuous arterial blood pressure will also be observed. If the blood pressure dropped to ≤90/60 mmHg, one recruitment maneuver was terminated in advance. And both groups of patients used the Dräger- or PB840-imported multifunctional ventilator. The treatment of primary disease and predisposing factors, fluid management strategies, antibiotics and glucocorticoids, nutrition, and metabolic support in the two groups of patients in the study were the same. The PaO2/FiO2 value improved by 51% 10 minutes after recruitment, and the median increased from 111 (IQR, 73-265) before recruitment to 170 (IQR, 102-340) (*P* < 0.01), the improvement of PaO2/FiO2 at 4 hours after recruitment and 12 hours after recruitment was 78% (*P* < 0.05) and 39% (*P* < 0.01), respectively, and the median PaO2/FiO2 at 4 hours after recruitment was 198 (IQR, 116-256). The median PaO2/FiO2 became 155 (IQR, 127-235) 12 hours after recruitment. Recruitment can reduce the accumulation of neutrophils in lung tissue, reduce the release of inflammatory factors, reduce pulmonary edema, and reduce pathological damage.

## 1. Introduction

Recruitment is a necessary complement to the low tidal volume lung protective ventilation strategy in ARDS. ARDS is an acute diffuse inflammatory alveolar injury induced by endogenous, exogenous, or compound injury factors and is one of the main causes of death in critically ill patients, with severe hypoxemia and respiratory distress as the main manifestations. At present, there is no effective drug treatment for ARDS, and it still stays at the level of supportive treatment such as mechanical ventilation and limited fluid replacement. Although most of the treatment measures are valuable in preclinical and early treatment, they have not shown the expected effect in the phase 2 and 3 clinical studies of ARDS. Possibly, the most important reason is the limitations of ongoing research on how to identify biological indicators relevant to ARDS criteria. Lung recruitment maneuvers can reduce the pulmonary recruitment of inflammatory cells, especially neutrophils in lung tissue, reduce the release of related inflammatory factors, reduce the changes in pulmonary edema and pathological damage in the model group, improve the oxygenation of patients, and shorten the lead time and reduce the fatality rate of patients.

The efficacy of lung recruitment is related to the etiology. The purpose of Longo et al. was to determine whether lung recruitment maneuvers could improve RV function by reventilating the lungs after CPB [1]. Chiou et al. performed air stacking with volume-preset ventilation or a manual resuscitator bag after all patients had stabilized vital capacity (reached a lifetime maximum) [2]. Liu et al. proposed a method to estimate lung recruitment characteristics from the static pressure-volume curve of the lung [3]. Sommerfield et al. discussed the clinical significance of recruitment maneuvers, the value of the use of recruitment maneuvers, and other techniques that can be used to reduce lung collapse [4]. The aim of Schults et al. was to identify and systematically review the quality of existing ETS CPG, especially with regard to NSI and RM usage [5]. However, their proposed lung recruitment manipulative therapy was not very effective.

Pulmonary exogenous ARDS is more effective than pulmonary endogenous ARDS. Yang et al. aimed to investigate the role of TNF-*α*, IL-1*β*, IL-9, and IL-15 cytokines in the pathogenesis of acute respiratory distress syndrome (ARDS) [6]. Toyama et al. established a mouse model of severe ARDS [7]. Wang et al. believed that neutrophil elastase (HNE) is a destructive enzyme that plays a crucial role in the pathophysiology of acute respiratory distress syndrome (ARDS) [8]. Shah et al. discussed the latest evidence for sedation management in ARDS patients [9]. Cannon et al. argued that early identification and minimization of further lung damage are critical for successful treatment of severe ARDS [10]. However, the ARDS method proposed by them is not very effective, and this paper introduces the lung recruitment maneuver to optimize it.

In this paper, the use of peripheral arterial monitoring of cardiac output technology can obtain reliable hemodynamic data through less trauma and timely detect hemodynamic changes and deal with them in time. Therefore, lung protective ventilation combined with lung recruitment is more conducive to lung gas exchange and lung protection and has little effect on hemodynamics. Once the alveoli are recruited, a higher level of PEEP is required to maintain the recruited alveoli open. There was no significant change in pairwise comparison between 20 minutes, 60 minutes, and 120 minutes after recruitment (*P* > 0.05).

## 2. Efficacy of Lung Recruitment in Patients with Acute Respiratory Distress Syndrome after Cardiopulmonary Bypass Surgery

### 2.1. Lung Recruitment

There are many lung recruitment maneuvers, and the most commonly used methods are controlled lung inflation, pressure control, PEEP (positive end expiratory pressure) incremental method, and sighing method. Among them, the PEEP incremental method is to complete the alveolar recruitment by gradually increasing the PEEP level and maintaining the ventilation pressure unchanged. For the lung image currently being processed, the cutting size of the top and bottom ends is calculated using the following formula [11]:

(1) $$\begin{array}{c} H_{u}=\frac{{H_{u}}^{\prime }}{h},\\ H_{d}=\frac{{H_{d}}^{\prime }}{h}. \end{array}$$

Among them, *H*_*u*_ and *H*_*d*_ are the top cutting length and bottom cutting length, respectively, and *h* is the height of the current lung image. The size cut by the left and right ends is calculated using the following formula [12]:

(2) $$\begin{array}{c} W_{l}=\frac{{W_{l}}^{\prime }}{w},\\ W_{r}=\frac{{W_{r}}^{\prime }}{w}. \end{array}$$

Among them, *W*_*l*_ and *W*_*r*_ are the cutting length at the left end and the cutting length at the right end, respectively, and *w* is the width of the current lung image [13].

For each lung image that needs to be processed, each pixel is traversed to calculate the gray value. The grayscale processing formula used is as follows:

(3) $$\begin{array}{c} gary\left(i,j\right)=\left(R_{ij}+G_{ij}+B_{ij}\right)/3. \end{array}$$

In the formula, *R*, *G*, and *B*, respectively, represent the lung pixel value of each layer channel [14].

However, in patients with poor response to recruitment, cardiac output (it refers to the amount of blood pumped by the left or right ventricle per minute) decreased during recruitment, while there was no significant change in patients with good response to recruitment. It is speculated that this may be related to the greater elasticity of the chest wall in patients with poor response to recruitment, resulting in higher pressure transferred to the thoracic cavity during recruitment. It is related to the local alveolar transpulmonary pressure difference. There are three main factors that affect the transpulmonary pressure difference: One is the closing pressure of the local alveoli, which is related to the surface tension of the alveoli, with an average of about 5 cmH_2_O. The second is the hydrostatic pressure, which increases gradually from the non-gravity-dependent region to the gravity-dependent region, ranging from 0 to 15 cmH_2_O. Alveolar surface tension refers to the extremely thin liquid layer distributed on the inner surface of the alveolar epithelium under normal conditions, forming an air-liquid interface with alveolar gas. It was confirmed by CT that most of the alveoli collapsed at PEEP 15 cmH_2_O. This pressure is similar to the hydrostatic pressure of ordinary people, so the hydrostatic pressure is most closely related to the opening and closing state of the alveoli and the setting of the corresponding PEEP level. In addition, the pressure was transmitted outside the lungs, such as increased intra-abdominal pressure and compression of the heart and mediastinum [15].

The joint probability distribution of the RBM is specified by the energy function:

(4) $$\begin{array}{c} P\left(v,h\right)=\exp\left(E\left(v,h\right)\right). \end{array}$$

The ARDS data normalization processing is

(5) $$\begin{array}{c} \hat{x}=\frac{x-E\left(x\right)}{\sqrt{Var\left(x\right)}}. \end{array}$$

Let the size of *R* be *l* × *l* × *n*, where *n* is the number of ARDS data feature maps [16]:

(6) $$\begin{array}{c} f_{i}={\left(\max-pool\right)}^{i}\times R_{i}. \end{array}$$

Among them, *R*_1_ and *R*_2_ are the central regions with sizes (*l*/2) × (*l*/2) × *n* and (*I*/4) × (*l*/4) × *n*, respectively.

The data is input in the input layer and starts to be passed to the last time, and finally, the final result of the network is obtained in the output layer, which is the last layer. The transmission relationship between them is as follows:

(7) $$\begin{array}{c} Z^{\left(l+1\right)}={XW}^{\left(l\right)}+b^{\left(l\right)},\\ \text{h}\left(\text{x}\right)=\text{f}\left(Z^{\left(l+1\right)}\right). \end{array}$$

In the formula, Z^(*l* + 1)^ represents the ARDS data output value, which represents the ARDS data output value of the *l* + 1th layer [17].

A total of 71 ARDS patients who met the inclusion criteria were included in this study, including 60 Han Chinese and 11 Uyghur patients, regardless of gender. The etiology of ARDS in all selected cases was cerebrovascular accident, 45 cases of cerebral hemorrhage (including 30 cases of traumatic cerebral hemorrhage and 15 cases of spontaneous cerebral hemorrhage), and 26 cases of cerebral infarction, a total of 71 patients. However, complications such as thoracic trauma, pneumothorax, lumbar fractures, and multiple fractures of limbs should be excluded. Apply propofol (a short-acting intravenous anesthetic) or midazolam to sedate the patient. Endotracheal intubation was connected to PB840 multifunctional ventilator for mechanical ventilation. A central venous catheter was placed in the internal jugular vein or subclavian vein, and a pressure sensor was connected. The radial artery cannula was connected to a pressure transducer and a Vigileo hemodynamic monitor. The selected patients will undergo 24 hours, 48 hours, and 72 hours of bronchoalveolar lavage when they board the machine, and the sediment will be counted and classified for inflammatory cells. The supernatant was placed in a -80°C freezer for MMP-9 (matrix metalloproteinase 9) assay. In addition, patients who underwent bronchoscopy for lung cancer were selected as the normal control group (normal group). The selected patients were Ia and Ib patients without mediastinal lymph node and pulmonary metastasis and with no history of chronic diseases such as heart, liver, and lung. The middle lobe or lingual lobe of the nondiseased lung was selected for bronchoalveolar lavage [18].

The patients were divided into lung recruitment group and conventional treatment group by random number permutation table method. When the patient's percutaneous oxygen saturation is less than or equal to 88% or the partial pressure of oxygen in the arterial blood gas is less than or equal to 55 mmHg, or the ventilator tube is disconnected during sputum suction or other accidents, all performed a CPAP (high pressure 40 ~ 45 cmH_2_O, PEEP 45 cmH_2_O) × 60 − second lung recruitment maneuver and then adjusted the ventilator parameters in the same way. During the process of lung recruitment, the changes of invasive continuous arterial blood pressure should be strictly observed. When the blood pressure dropped to ≤90/60 mmHg, one recruitment maneuver should be terminated in advance. Arterial blood pressure refers to the lateral pressure (pressure) of blood on the aortic wall per unit area, which generally refers to the blood pressure in the aorta. The general condition of the patient has improved, the consciousness is clear, and the ability to expectorate sputum is strong. When FiO_2_ reduced to 40%, keep SPO_2_ ≥ 88 ~ 95% or PaO_2_ ≥ 55 ~ 80 mmHg for 24 hours, switch to PSV+PEEP (adjust the breathing frequency of mechanical ventilation to 0), adjust the inspiratory time to 1.5~1.6 seconds, and gradually reduce PEEP to 5 cmH_2_O. Then gradually reduce the support pressure to 5~7 cmH_2_O. After 5 ~ 7 cmH_2_O × 5 cmH_2_O is set for 2 hours, the patient can be off-line with stable breathing and circulation, followed by sequential noninvasive mechanical ventilation. The application of sedation in the two groups was alternately applied diprima and midazolam, and the sedation score was maintained within 72 hours of the Ramsay (The most widely used sedation score in clinical practice, simple and practical) score of 3-4. Both groups of patients used the Dräger- or PB840-imported multifunctional ventilator. The treatment of primary diseases and predisposing factors, fluid management strategies, antibiotics and glucocorticoids, nutritional and metabolic support, and other application principles of the two groups of patients are the same [19, 20].

After confirming that there is no abnormality in the skin, select the skin on the head, neck, and side chest wall where electrodes are to be placed, and wash the selected skin with warm water and alcohol gauze. Before determining the skin of the sticking site, make sure that the skin where the electrode pads are placed is clean. If there is dead skin and hair, completely remove the oily secretions and dead skin cells from the corresponding part of the patient. If there is iodophor in the skin area, be sure to completely deiodine with alcohol, and thoroughly dry the skin before installing the electrode pads. Pay attention to whether there is any abnormality in the waveform of the noninvasive cardiac output monitoring (a noninvasive way to obtain hemodynamic data by measuring blood flow instead of blood pressure) [21]. Once the quality of the outgoing signal is poor and the parameter display is incomplete, people should first check whether the position of the electrode is in the correct position and ensure that the electrode pad is tightly attached to the patient's skin. There is no looseness or poor contact between them, and at the same time, confirm whether the connection of various wires is abnormal. If it is confirmed that the connection is correct, the contact is good, the waveform does not appear, or the waveform is abnormal, it is necessary to replace a new set of electrodes. The lung recruitment process is shown in Figure 1 [22].

### 2.2. Cardiac Surgery with Cardiopulmonary Bypass

In view of the characteristics of lung injury during CPB, perfusion of protective solution or oxygenated blood from pulmonary artery during CPB has become a direction of lung protection research. In short, during cardiopulmonary bypass, according to a certain perfusion method, the protective fluid or blood is perfused to the lungs through the pulmonary artery cannula. It has been found in theory and practice that during cardiopulmonary bypass, pulmonary artery perfusion with protective fluid may reduce the degree of lung tissue damage caused by ischemia and inflammatory response, thereby protecting lung function. During cardiopulmonary bypass and pulmonary ischemia, pulmonary artery perfusion with oxygenated blood or crystalloid as protective fluid can provide the necessary oxygen supply or help to enhance the stability of vascular endothelial cells, maintain satisfactory colloid osmotic pressure, protect alveolar surfactant, and prolong lung ischemia tolerance time. Adding an appropriate amount of active substances to the protective solution can further promote the protection of pulmonary blood vessels: For example, prostaglandin E1 can help dilate pulmonary blood vessels and protect the stability of cell membranes. L-arginine (an organic compound) can provide the necessary substrate for NO synthesis, which is conducive to the maintenance of vascular tone and patency. Anisodamine helps maintain vascular smooth muscle activity and relieve vasospasm. Methylprednisolone helps relieve inflammation and maintain cell membrane stability. Acid-base buffers help to neutralize hypoxic metabolites and maintain vascular homeostasis [23].

The ARDS variance at position (*i*, *j*) in the image at time *t* is calculated as follows:

(8) $$\begin{array}{c} \varepsilon_{ij}^{t}={\left(\sigma_{ij}^{t}I_{ij}^{t}-G_{ij}\right)}^{2}. \end{array}$$

The ARDS Gaussian formula is as follows [2]:

(9) $$\begin{array}{c} G\left(x,y,\delta \right)=\frac{1}{2\delta^{2}}e^{\left(x^{2}+y^{2}\right)}. \end{array}$$

The main flow of change detection is shown in Figure 2. Different types of medical images have different processing methods in the preprocessing stage. For medical images, in order to obtain more accurate and higher resolution images, it is necessary to remove irrelevant parts. This process includes image registration and denoising. The quality of image recognition is related to the amount of feature extraction. For images, especially medical images, the traditional input method is to use pixel values as input, so the image will be divided into pixels, numbers like 0 and 1. For the classifier, this shallow signal cannot be recognized, so classification is difficult. If the high-dimensional features of the image are used, in addition to the pixel points as the input, the relationship between the pixels must be used as the input. At this point, the classifier can classify the image through the classification rules (a subcategory of the global assortment can be a global assortment, a customer-specific assortment, or a mix of the two). And this process is called feature extraction. In addition to the feature extraction stage, it is also necessary to analyze the features. The general process of feature analysis is to use the clustering algorithm or the deep neural network algorithm to extract the features in the image and then analyze the extracted features according to the process of finally generating a binary image. In this paper, after extracting features, a deep belief network is used for analysis. Clustering is a widely used exploratory data analysis technique. After feature analysis, the results of change detection need to be evaluated. In the binarized image, the black area represents the area that has not changed in the change detection, and the white area represents the area that has changed [24].

Sensitivity represents the probability that the patient's lesion is correctly detected, and its expression is as follows:

(10) $$\begin{array}{c} \text{Sensitivity}=\frac{\text{TP}}{\text{F}}. \end{array}$$

The Kappa coefficient represents a degree of closeness. If the real map of the lung unit is similar to the network output map, the Kappa value is closer to 1, and vice versa, the Kappa value is closer to 0. Its expression is as follows:

(11) $$\begin{array}{c} \text{Kappa}=\frac{P-\text{PRE}}{1-P}. \end{array}$$

The formula for PRE is as follows:

(12) $$\begin{array}{c} \text{PRE}=\frac{\left(\text{TP}+\text{F}\right)\times \text{Mc}+\text{FN}\times \text{Mu}}{\text{TP}+\text{F}+\text{FN}}. \end{array}$$

### 2.3. Acute Respiratory Distress Syndrome

Since ARDS is a form of pulmonary edema, fluid management is an essential aspect of its treatment. Fluid overload is associated with poor prognosis in critically ill patients, requiring aggressive fluid resuscitation in the early stages of resuscitation and organ failure. Subsequent tapering of fluid load (so-called reverse volume resuscitation) was done after hemodynamic stabilization, either spontaneous or induced. Fluid load can cause or exacerbate AKI through a variety of mechanisms. Lung injury due to fluid overload mirrors that caused by intravenous fluid infusion. Rapid fluid infusion in healthy volunteers can cause interstitial pulmonary edema. Patients with sepsis who receive fluid bundle therapy in the early resuscitation phase will experience decreased oxygenation and worsening lung injury scores. Subsequent studies have demonstrated that the open infusion strategy can easily lead to fluid accumulation, especially in the case of severe infection and capillary leak syndrome (a sudden, reversible symptom of capillary hyperpermeability), which can lead to increased intracapillary hydrostatic pressure. Furthermore, on the basis of osmotic pulmonary edema, interstitial pulmonary edema with increased hydrostatic pressure was developed. In mechanically ventilated ICU patients, the addition of immunomodulatory nutrients to enteral feeding did not reduce the incidence of infection. There are no direct comparative studies of how to choose the optimal sedation or depth of sedation in ARDS. In general, patients should be lightly sedated without pain, and benzodiazepines should be avoided as much as possible. Early deep sedation is associated with increased mortality in mechanically ventilated patients. In contrast, early rehabilitation exercise is beneficial to improve the prognosis of mechanically ventilated ARDS patients. The fusion formula is as follows:

(13) $$\begin{array}{c} F=concat\left(F_{lr}\right). \end{array}$$

Pearson's correlation coefficient of ARDS patients' condition is as follows:

(14) $$\begin{array}{c} PLCC=\frac{\sum_{i=1}^{N}\left(y_{i}-{\hat{y}}_{i}\right)\left(y-\hat{y}\right)}{\sqrt{\sum_{i=1}^{N}{\left(y_{i}-y\right)}^{2}{\left({\overset{\wedge }{y}}_{i}-\overset{\wedge }{y}\right)}^{2}}}. \end{array}$$

The Spearman correlation coefficient of the condition of ARDS patients is as follows:

(15) $$\begin{array}{c} Soc=1-\frac{\sum_{i=1}^{N}\left(v_{i}-p_{i}\right)}{N^{2}}. \end{array}$$

In this paper, the mean square error (MSE) function is used as the loss function, and the calculation formula is as follows.

(16) $$\begin{array}{c} s=\overset{N}{\underset{i=1}{\sum }}{\left(\frac{1}{n}\right)}^{2\left(y_{i}-q_{i}\right)}. \end{array}$$

Among them, *y*_*i*_ is the ground-truth label of the lung image, and *q*_*i*_ is the subjective quality value of the lung image.

About 50% of the patients who meet the diagnostic criteria of ARDS were autopsied, but no diffuse alveolar damage was found as a specific pathological manifestation. These patients may have some coexisting diseases. However, in most positive trials so far, the improved prognosis in the intervention group is the result of less ventilator-related injury. All mechanically ventilated patients are at risk of ventilator-associated lung injury, so the heterogeneity of ARDS cases collected should be minimized. If a specific biological indicator is studied as a therapeutic target, its heterogeneity may become more important; otherwise, its ability to detect possible effects may be reduced. In the case of individualized treatment of ARDS, the discovery of effective biomarkers can not only identify special populations but also help to identify specific treatment measures. Polymorphonuclear leukocytes play an important role in the pathogenesis of ALI/ARDS and are the main inflammatory cells that mediate local inflammatory damage to the lung. In the early stage of ARDS, cytokines have chemotactic and activation effects on neutrophils (neutrophils in the lung parenchyma are rare under normal circumstances), neutrophils are recruited and migrate into the capillaries of lung tissue, causing damage to pulmonary capillary endothelial cells, pulmonary interstitium, and alveolar epithelial cells, destroying the barrier function of pulmonary vascular endothelium and causing permeability pulmonary edema. ARDS is a group of syndromes with diverse etiologies and similar clinical manifestations, characterized by heterogeneous pulmonary infiltrates. Mechanical ventilation is a compromise ventilation method of last resort for the heterogeneous lung consolidation in ARDS. However, the resulting alveolar collapse, the repeated opening and trapping of lung tissue (shear force), and the release of biological mediators further lead to intrapulmonary and extrapulmonary damage cannot be ignored. Common symptoms of pulmonary infiltrates include cough, expectoration, fever, fatigue, night sweats, and hemoptysis. Therefore, lung recruitment can not only open the collapsed alveoli and increase the lung capacity but also reduce the shear force damage caused by the periodic opening of the lung tissue in the collapsed area and the normal area. It can also avoid lung damage caused by hyperventilation of some alveoli in the “baby lung” of ARDS. So as to improve ventilation and ventilation function, reduce inflammation, and improve prognosis.

ARDS symptom severity is calculated as follows:

(17) $$\begin{array}{c} ARDS=\overset{M}{\underset{i=0}{\sum }}\overset{N}{\underset{j=0}{\sum }}x\left(i,j\right). \end{array}$$

There are many methods of lung recruitment, mainly including controlled lung inflation, pressure control, and PEEP increments. In this paper, the individualized PEEP incremental method is used, because this method is mainly to gradually increase the PEEP level and can complete the alveolar recruitment under the condition of maintaining the ventilation pressure unchanged. The advantage of this method is that the whole process takes a short time, and it can maintain a basically constant tidal volume under the condition of constant ventilation pressure, which reduces the risk of volutrauma. It is one of the more commonly used research methods. When the balance of the two is disrupted by various etiologies, there is out of balance, which leads to systemic inflammatory response (SIRS). When a systemic inflammatory response occurs, under the action of the cascade effect of various inflammatory mediators released by polymorphonuclear leukocytes (PMN) and mononuclear macrophages in the lung tissue, the inflammation occurs. It leads to the damage of lung epithelial cells and vascular endothelial cells, affects various enzyme activities of tissue cells, and causes the imbalance of sodium and water transport system inside and outside the interstitial space. It greatly reduces the production of surfactants needed to promote alveolar recruitment and allows a large amount of protein-rich colloid fluid to enter the lung tissue, which affects the normal absorption and exchange of normal lung tissue fluid. It eventually leads to acute pulmonary edema, the formation of the hyaline membrane of the lung, and the trapping of the alveoli, which affect the gas exchange of the body, both of which are the basis for the body to produce hypoxemia. In addition, in the systemic inflammatory response, inflammatory factors such as platelet activating factor and arachidonic acid metabolite cannot be ignored and play an important role in the development of the disease. RDS has onset, acute onset, and rapid progress. Currently, the treatment measures for RDS are mainly comprehensive treatment in multiple aspects, mainly including: The first is the treatment of the primary disease, which is the fundamental treatment, as well as respiratory support to improve the patient's hypoxemia, protection of the function of important organs in the body, and appropriate targeted drug treatment. Due to the rapid progress of the patient's condition, it is particularly important to emphasize early intervention.

## 3. Therapeutic Efficacy of ALI-ARDS Patients

pH value and PCO2 recruitment stage did not change significantly. The means of PO2 and PO2/FiO2 (short for fraction of inspiration O2, which is the fraction of oxygen concentration in the inhaled air) are not all the same in each group, and the *q* test is used for pairwise comparison. The results showed that the PO2 and PO2/FiO2 groups increased at 20 minutes, 60 minutes, and 120 minutes after recruitment, compared with those before recruitment, with statistical significance (*P* < 0.05). However, there was no significant change in pairwise comparison between 20 minutes, 60 minutes, and 120 minutes after recruitment (*P* > 0.05). The changes in blood gas indexes are shown in Table 1.

Among them, *Pplat* and *Pm* were significantly higher at 60 minutes after recruitment and 120 minutes after recruitment, and the difference was significant (*P* < 0.05). There was no difference between the other groups (*P* > 0.05). *Pplat* and *Crs* were significantly increased at 20 minutes, 60 minutes, and 120 minutes after recruitment, and the differences were significant. There was no significant difference between the other groups (*P* > 0.05). The respiratory mechanics indexes before and after recruitment are shown in Table 2.

Taking the prerecruitment arterial blood gas index as the control, the PaO2/FiO2 value was improved by 51% 10 minutes after the recruitment, and the median increased from 111 (IQR, 73-265) before recruitment to 170 (IQR, 102-340) (*P* < 0.01). The improvement of PaO2/FiO2 at 4 hours after recruitment and 12 hours after recruitment was 78% (*P* < 0.05) and 39% (*P* < 0.01), respectively. The median PaO2/FiO2 4 hours after recruitment was 198 (IQR, 116-256). The median PaO2/FiO2 at 12 hours after recruitment was 155 (IQR, 127-235). The change of the influence of PaO2/FiO2 is shown in Figure 3.

This paper found that the heart rate (HR) at the selected time points before and after lung recruitment was not significantly different from that before recruitment. The mean arterial pressure (MAP) increased to 8, 10 cmH2O (*P* < 0.01), and 12 cmH2O (*P* < 0.05) in the PEEP during the recruitment process compared with those before recruitment. The mean arterial pressure (MAP) decreased to 6, 10 cmH2O (*P* < 0.01), 8, and 12 cmH2O (*P* < 0.05) in the process of recruitment, and the PEEP was also significantly different from that before recruitment. During the implementation of lung recruitment, none of the patients terminated recruitment due to blood pressure fluctuations, so the difference before and after has no clinical significance. The changes of heart rate and mean arterial pressure when PEEP were downregulated and raised during recruitment are shown in Figure 4.

The time from the onset of ARDS to the onset of the primary disease was 20.76 ± 28.90 hours, and the 25th, 50th, 75th, 90th, and 95th percentiles were 1, 3.48, 72, and 72 hours, respectively. ARDS occurred 29.0 ± 37.51 hours after sepsis (systemic inflammatory response syndrome caused by the invasion of pathogenic microorganisms such as bacteria into the body), 21.47 ± 30.77 hours after pneumonia, and ARDS was 9.0 ± 2.0 hours from the onset of other primary diseases. There was no statistical significance among the three (*F* = 2.073, *P* = 0.166). The time from the onset of ARDS to the onset of other primary diseases was shorter than that from the onset of pneumonia and sepsis.  Figure 5 shows the statistics of the time between the onset of ARDS and the onset of the primary disease.

A total of 393 cases of pneumonia were treated in PICU, and 15 cases of ARDS occurred; the incidence rate was 3.8%, 95% confidence interval (2.3%, 5.1%). ARDS occurred in 3 of 90 patients with sepsis, the incidence rate was 3.3%, 95% confidence interval (2.2%, 5.0%). The etiology distribution of ARDS is shown in Figure 6.

There was no significant difference in cardiac coefficient (CI) and peripheral vascular resistance index (SVRI) one hour before and after lung recruitment (*P* > 0.05), but there were significant differences in SPO2 and PaO2/FiO2 (*P* < 0.05). The changes of blood flow dynamics and oxygenation index before and after lung recruitment in the supine position of the patients are shown in Table 3.

Comparison of the tendency position of heart rate (HR), CVP, mean arterial pressure (MAP), cardiac coefficient (CI), peripheral vascular resistance index (SVRI), and stroke volume index (SVI) before and 1 hour after mobilization does not have statistical significance (*P* > 0.05). The difference between pO2 and PaO2/FiO2 was statistically significant (*P* < 0.05). The changes of blood flow status and oxidative index before and after lung recruitment in the prone position are shown in Table 4.

There was no significant change in hemodynamic parameters before and after mobilization in the supine position and before and after the mobilization in the prone position (*P* > 0.05). The comparison of hemodynamic parameters is shown in Table 5.

In the SI group, MAP also decreased significantly during RM. In the PCV (pressure control ventilation) group, MAP (mean arterial pressure) also fluctuated at the beginning of RM. However, the amplitude and duration of the fluctuations were smaller than those in the SI (controlled inflation, sustained inflation) group. The comparison of PCV and SI is shown in Figure 7.

Mean pulmonary arterial pressure (MPAP) and pulmonary capillary wedge pressure (PCWP) were significantly increased after lung injury, but PCWP < 18 mmHg. Central venous pressure (CVP) did not change much before and after lung injury. The changes of MPAP and PCWP are shown in Figure 8.

There are many causes of acute respiratory distress syndrome (ARDS) in patients; no matter what kind of cause, the main pathophysiological changes are the same. As the disease progresses, the patient often feels labored to breathe, the respiratory rate increases, and the blood gas indicators are mostly hypoxemia with hyperventilation, respiratory alkalosis caused by excessive carbon dioxide excretion, tightness in the chest, and cyanosis of the skin and lips at the extremities. Due to the lack of oxygen in the brain, it is often accompanied by disturbance of consciousness, and at the same time, there is a decline in orientation and judgment. The chest X-ray of both lungs showed interstitial pulmonary edema, and general oxygen inhalation therapy was given for dyspnea, but the symptoms could not be relieved. With the progress of the disease to the later stage, the clinical collectively known as “big white lung” may appear. Patients with persistent hypoxemia can only be relieved by mechanical ventilation, and ventilator-related lung injury may exist when conventional ventilator-assisted ventilation is used. In order to reduce and minimize lung injury, the current ventilation strategy has been improved, the main purpose is to maintain the most basic oxygenation state of the patient, use the minimum tidal volume, and minimize or even avoid ventilator-related lung injury. The effects of PtpPEEP on hemodynamics and oxygenation are shown in Figure 9.

The effect of PtpPEEP value on ARDS patients is shown in Figure 10. Compared with the ground state, the Cst increases significantly when the PtpPEEP values are 3 cmH2O, 6 cmH2O, and 9 cmH2O.

## 4. Conclusion

The lung recruitment maneuver is a new and controversial treatment method beyond the conventional ventilation mode. The basic method is to break through the forbidden area of traditional ventilation mode, continuously or intermittently increase the pressure across the pulmonary artery, and increase the distribution of gas in the alveoli. All the selected patients were firstly treated with mechanical ventilation in the supine position, the ventilation mode was synchronized intermittent mandatory ventilation, and lung recruitment was performed one hour after the basal ventilation. One hour after lung recruitment, after a 15-minute washout period, the patient's position was changed to the prone position. Immediately after basal ventilation was performed for one hour, lung recruitment was performed. The recruitment maneuver was the same as the supine position, and the interval between the two positions was at least two hours. The main purpose of using the washout period is to minimize the effect of the supine position recruitment on the prone position before recruitment, and there is a superposition effect, which affects the results of the study. In diseases with low lung compliance, the most important role of ARM is to equalize the pressure distribution of the lung parenchyma in heterogeneous lesions. Therefore, ARM can avoid excessive expansion of normal alveoli (volumetric lung injury) and collapse of partially ventilated alveolar units (atelectasis lung injury) while resuscitating nonventilated alveoli. Recruitment can open more alveoli and allow the lungs to perform more gas exchange at lower respiratory pressures. Future work should explore the effect mechanism of ARDS duration on lung recruitment.

## Figures and Tables

**Figure 1:** Lung recruitment process.

**Figure 2:** Main flow of change detection.

**Figure 3:** Changes in the influence of PaO2/FiO2.

**Figure 4:** Changes in heart rate and mean arterial pressure when PEEP was downregulated and raised during recruitment.

**Figure 5:** Time from onset of ARDS to onset of primary disease.

**Figure 6:** ARDS etiology distribution.

**Figure 7:** Comparison of PCV and SI.

**Figure 8:** Changes in MPAP and PCWP.

**Figure 9:** Effects of PtpPEEP on hemodynamics and oxygenation.

**Figure 10:** Effect of PtpPEEP value on ARDS patients.

**Table 1:** Changes in blood gas indexes.

Blood gas index	Before recruitment	After recruitment 20 min	After recruitment 60 min	After recruitment 120 min
pH	4.80	5.38	6.14	6.23
PCO2 (mmHg)	32.33	33.13	34.78	39.31
PO2 (mmHg)	59.64	67.29	72.98	73.56
PO2/FiO2	117.49	123.82	149.88	161.49

**Table 2:** Respiratory mechanics parameters before and after recruitment.

Respiratory mechanics	Before recruitment	After recruitment 20 min	After recruitment 60 min	After recruitment 120 min
PIP (cmH2O)	19.23	18.35	17.22	17.20
*Pplat* (cmH2O)	17.08	16.82	16.50	16.21
*Pm* (cmH2O)	17.58	17.26	17.21	17.20
*Crs* (cmH2O)	36.71	36.92	37.19	37.72

**Table 3:** Changes of blood flow dynamics and oxygenation index before and after lung recruitment in the supine position.

Variable	Before recruitment	1 h after recruitment
HR (times/min)	83.4 ± 4.2	84.0 ± 4.6
CVP (cmH2O)	63 ± 2.6	6.4 ± 2.8
MAP (mmHg)	63.0 ± 3.4	64.2 ± 3.6
CI (L/min)	3.6 ± 0.6	3.6 ± 0.3

**Table 4:** Changes in blood flow status and oxidative index before and after lung recruitment in prone position.

Variable	Before recruitment	1 h after recruitment
HR (times/min)	73.3 ± 3.1	73.0 ± 3.5
CVP (cmH2O)	53 ± 1.5	5.3 ± 1.7
MAP (mmHg)	53.0 ± 3.3	53.1 ± 3.5
CI (L/min)	3.5 ± 0.5	3.5 ± 0.3

**Table 5:** Comparison of hemodynamic parameters.

Variable	Supine position P	Prone position P
HR (times/min)	0.734	0.447
CVP (cmH2O)	0.873	0.742
MAP (mmHg)	0.834	0.847
CI (L/min)	0.742	0.774

## Data Availability

Data sharing is not applicable to this article as no datasets were generated or analysed during the current study.
